# Research Progress on the Effect of Traditional Chinese Medicine on Signal Pathway Related to Premature Ovarian Insufficiency

**DOI:** 10.1155/2022/7012978

**Published:** 2022-09-14

**Authors:** Yidi Wang, Xiuxiang Teng, Jun Liu

**Affiliations:** ^1^Capital Medical University, Beijing 100069, China; ^2^Beijing Hospital of Traditional Chinese Medicine, Capital Medical University, Beijing 100010, China

## Abstract

The occurrence and development of premature ovarian insufficiency involves the abnormality of multiple signal pathways. It is a complex disease. Traditional Chinese medicine affects the relevant factors of the occurrence and development of premature ovarian insufficiency (granulosa cell apoptosis, ovarian blood supply, ovarian reserve, ovarian oxidative damage, gap junction, ovarian fibrosis, follicular development, follicular atresia, and other biological processes) by regulating a variety of signal pathways, thus playing the role in antioxidant stress, prevention and treatment of chemotherapy side effects, protection of ovarian function, control of aging, and improvement of ovarian reserve function. The research shows that the research on the related pathways of traditional Chinese medicine in the treatment of premature ovarian insufficiency has been quite extensive. Based on the search of the domestic and foreign literature, it is found that Yulinzhu and Xianziyizhen capsule and ginsenoside Rg_1_ can promote the proliferation and differentiation of granulosa cells, inhibit apoptosis, and reduce follicular atresia by affecting the PI3K/Akt/mTOR signal pathway; Guiluo's Anzang decoction, Kuntai capsule, and Yangyin Shugan granule can maintain the balance between pro-apoptotic protein and anti-apoptotic protein through the Bax/cytc/caspase-3 pathway to improve ovarian reserve function; Bushen Jianpi recipe can control cell apoptosis and promote the proliferation and development of ovarian granulosa cells by regulating the MAPK signal pathway; Siwu mixture and Zuo Gui pill can regulate the TGF-*β*/Smads signaling pathway to promote the recruitment of primordial follicles, promotes follicular development, inhibits follicular atresia, and regulates ovarian function; Erxian decoction, Yiqi Yangrong Fujing formula, and Cistanche deserticola can antagonize the inflammatory symptoms of premature ovarian failure, promote the secretion of relevant vascular growth factors, and enhance the ovarian reserve function through the NF-KB signal pathway; Bushen Culuan decoction can promote damage repair and protect normal ovarian cells through antioxidant stress. The above summary aims at providing reference for the in-depth study of traditional Chinese medicine in the treatment of premature ovarian insufficiency and inspiring new diagnosis and treatment ideas.

## 1. Introduction

Premature ovarian insufficiency (POI) is defined as a decline in ovarian function that occurs in women before the age of 40 years, resulting in abnormal menstruation, increased FSH levels, decreased estrogen volatility, and decreased fertility. Clinical female patients will have hot flashes, sweating, vaginal dryness, mood changes, and fertility difficulties. POI also increases a woman's risk of osteoporosis, and cardiovascular and cognitive disorders, according to related studies. Thus, the decline of ovarian function seriously reduced the patient's quality of life. At present, the incidence of POI is 1%∼65% and has a tendency to increase. Its pathogenesis is also not clear in the existing guidelines, and expert consensus suggests that treatment with hormone replacement therapy is given priority and can effectively relieve the clinical symptoms, but the side effect is more apparent, such as patients with uterine using estrogen therapy may increase the risk of endometrial cancer. Estrogen and progesterone can increase the risk of ovarian cancer [1]. Therefore, it is important to find nonhormone replacement therapy.

Traditional Chinese medicine treatment is characterized by syndrome differentiation and treatment, which varies from person to person and has few side effects. In traditional Chinese medicine, POI can be classified into “amenorrhea,” “infertility,” and “blood depletion” [2]. The pathogenesis is mostly due to the deficiency of Yin and blood in the kidney, in combination with liver depression, spleen deficiency, dampness and heat, vein stasis, etc. The treatment of TCM is mainly based on the principles of nourishing Yin and blood, warming the kidney Yang, relieving liver depression, strengthening the spleen, benefiting Qi, activating blood stasis, , and focusing on comprehensive treatment by identification. With the continuous research and excavation of TCM, more and more reports point out that TCM can treat POI through multiple pathways and targets. On this basis, the author collated the domestic and foreign literature in recent years to summarize the pathways of TCM in the treatment of POI and to provide a basis for clinical use.

## 2. PI3K/Akt Signaling Pathway

Phosphatidylinositol 3-kinase (PI3K) signaling pathway is the basic signaling pathway in animals, playing an indispensable role in cell growth, proliferation, survival, migration, metabolism, and apoptosis [3]. Studies in recent years have revealed that the PI3K/Akt pathway also plays an important role in premature ovarian insufficiency. For example, the PI3K/Akt/mTOR signaling pathway has a regulatory role in the HPG axis [4], and the activated Akt pathway further causes a cascade reaction of signaling pathway, and phosphorylated Akt can phosphorylate a series of downstream target proteins. It includes FOXO3a (antiproliferation and apoptosis), BAD (a pro-regulatory member of the Bcl-2 family, involved in cellular mitochondrial regulatory pathways), mTOR (which controls protein biosynthesis and regulates cell growth), and P27 (which maintains primal follicular reserves).

### 2.1. PI3K/Akt/mTOR Signaling Pathway

The complex TSC1/2 is both an oncogene and a major inhibitor of mTORC1. Elevated AKT expression promotes the separation of the complex TSC1/2, and the dissociation of the two releases the inhibition of mTORC1 and activates mTORC1, thus allowing the activation of the mTOR signaling pathway. The mTOR activation can inhibit autophagy and thus promote cellular senescence.

A nonrandomized noninferiority controlled study [5] conducted by Teng Xiuxiang et al. found that after treatment with Yulinzhu plus reduction in the treatment group, compared to the control group treated with estradiol valerate tablets plus progesterone capsules, the treatment group had significantly better overall efficacy (61.54%) and TCM evidence efficacy (49.45%), and serum FSH, LH, and *E*_2_ were significantly improved compared to the control group. One study reported [6] that after immune POI mice were given the Chinese herbal medicine Yulinzhu for 6 weeks, Akt protein expression was significantly increased and TSC1 and TSC2 protein expression was significantly decreased in each administration group. RheB, P-s6k1, and P-4E-BP1 protein expressions were elevated, with P-4E-BP1 being the most significantly elevated, ROS and MDA were significantly elevated, and GSH-Px and SOD were significantly decreased, indicating that Yulinzhu inhibits microenvironmental oxidative stress by regulating the TSC/Akt signaling pathway.

A randomized controlled trial [7] conducted by Lin Xiuqin found that the total response rate of Jiajian Guishen pill combined with estradiol valerate tablets and progesterone capsules in the observation group and estradiol valerate tablets and progesterone capsules in the control group was 93.33% and 70%, respectively, with statistically significant differences. In a study by Kong [8], it was found that Jiajian Gui Shen pill was able to increase the number of follicles at all levels in the ovaries of VCD-induced mice, reduce atretic follicles, improve serum sex hormone levels, and also improve ovarian function possibly by upregulating PI3K, Akt, mTOR mRNA, and protein expression levels.

Huang et al.[9] showed that the Xianzi Yizhen capsule was able to increase Ki-67, Akt, and PI3K protein expression and concluded that the mechanism of improving ovarian function might be related to increased PI3K/Akt pathway activity and cell proliferation status in ovarian cells, which increased the content of primordial follicles, secondary follicles, and sinusoidal follicles and decreased the content of atretic follicles.

Ginsenoside Rg1 is an important pharmacologically active component of ginseng, which has the ability to promote the secretion of estrogen and luteinizing hormone (LH). Liu et al.[10] observed that ginsenoside Rg1 can effectively inhibit the expression of PI3K, Akt, mTOR, and S6k proteins compared to the high expression of PI3K, Akt, mTOR, and S6k proteins in aging tissues, indicating that ginsenoside Rg1 can negatively regulate the PI3K/Akt/mTOR signaling pathway and activate autophagy in ovarian tissues, thereby inhibiting the onset of aging and prolong lifespan.

Icariin is a flavonoid extracted from Epimedium, which has phytoestrogen-like effects. Dong [11] found that Epimedium phosphorylated the activation of PI3K/Akt/mTOR signaling pathway-related proteins during the development of chemotherapy-injured POF, inhibited oxidative stress to reduce tissue apoptosis, and improved chemotherapy-injured POF in mice.

Thus, the PI3K signaling pathway not only regulates the growth of oocytes, regulates the survival and development of primordial follicles, and promotes the proliferation and differentiation of granulosa cells, but also inhibits apoptosis, which is crucial for the normal development and physiological function of ovaries.

### 2.2. Bax/CytC/Caspase-3

Bcl-2 and Bax are a pair of anti-apoptotic proteins that are antagonistic to each other. Bcl-2, which is mainly found in the outer mitochondrial membrane and part of the endoplasmic reticulum, can play its role in inhibiting apoptosis by blocking the release of mitochondrial CytC and then preventing the activation of caspase apoptosis protein. When cells receive apoptotic signals, Bax translocates into the mitochondria and exerts its pro-apoptotic effect by promoting the release of CytC in large amounts and further initiating the caspase cascade reaction. Whether the cells continue to survive or go to death depends to some extent on the ratio of Bcl-2 to Bax.

Yi-Hui observed [12] that Gui Luo's Anzang decoction could increase Bcl-2 protein expression and decrease Bax protein expression in the ovary, reduce granulosa cell apoptosis, and increase granulosa cell secretion.

A meta-analysis of a randomized controlled trial [13] conducted by Liu et al. showed that the total effective treatment rate of Kuntai capsules combined with hormonal therapy for POF was significantly better than that of hormonal therapy alone (OR = 3.76, 95% CI [2.65, 5.35], *P* < 0.00001). In an experiment, Geng [14] observed that the Kuntai capsule could improve ovarian reserve by downregulating the levels of FSH and LH, stimulating *E*_2_ secretion, regulating the Bcl-2/Bax ratio among Bcl-2 family protein members, and upregulating the expression of Bcl-2 and Bcl-xl proteins versus downregulating the expression of Bax and Bad proteins to maintain the balance between pro-apoptotic and apoptosis-inhibiting proteins.

Wang [15] found that Yangyin Shugan granule could regulate the expression levels of apoptosis-related proteins in ovarian tissues, increasing the expression of Bcl-2 protein and decreasing the expression of Bax and caspase-3 proteins, thus inhibiting apoptosis.

A systematic evaluation [16] conducted by Hu et al. showed that the efficacy of Zuo Gui pill combined with western artificial cycles was superior to treatment with western artificial cycles alone for premature ovarian failure, with significant advantages in the combined group in terms of improved menstrual rates and improved values of serum FSH, and Wang [17] and Gao [18] found through experiments that Zuo Gui pill could increase the level of Bcl-2 mRNA and decrease the level of Bax, and Bcl-2>Bax, concluding that the kidney Zuo Gui pill may inhibit chemotherapy-induced granulosa cell apoptosis by affecting the expression levels of apoptotic factors Bcl-2 and Bax, and thus play a role in protecting ovarian function.

### 2.3. FOXO3 Transcription Factor-P27/Bim

FOXO3 is an important transcription factor downstream of the PI3K/Akt pathway. When the Akt pathway is inhibited, dephosphorylated FOXO3 enters mostly into the nucleus and accelerates cell regulation. FOXO3 together with RUNX3 binds to the Bim gene in order to activate Bim and thus induce cell regulation.

A randomized controlled trial [19] conducted by Xiao et al. found that in POI, the clinical efficacy of Erxian decoction (95.00%) was significantly better than that of the estradiol valerate combined with the progesterone group (77.50%). In an experiment, Zhao [20] observed that Erxian decoction had a protective effect on cisplatin-injured ovarian granulosa cells. On the one hand, it may be that Erxian decoction exerts a pro-proliferative effect by affecting the granulosa cell cycle phase, promoting the transformation of granulosa cells from *G*_*0*_ to S phase, decreasing the proportion of *G*_0_ phase cells, increasing the ratio of S phase cells, and improving the proliferation index; on the other hand, it may be that Erxian decoction exerts an antiregulatory effect by decreasing the rate of cisplatin-induced granulosa cell apoptosis. And it was further found that the protective effect of Erxian decoction on cisplatin-induced ovarian granulosa cells might be achieved by regulating the expression of FOXO3a and its downstream target proteins. Thus, Erxian decoction can downregulate the expression of FOXO3a in cisplatin-injured granulosa cells, which in turn downregulates the expression of cell cycle blocker protein P27^kip1^ and pro-apoptotic protein Bim, thus promoting granulosa cell proliferation and inhibiting granulosa cell regulation.

Yang [21] found that the intervention of Zuo Gui pill in the experiment may affect the p-Akt-to-Akt ratio by upregulating the p-Akt level on the PI3K/AKT pathway, as well as reducing FOXO3a protein expression, which in turn effectively inhibits granulosa cell damage and prevents premature follicular failure and atresia in order to protect ovarian function.

In addition, Yangyin Shugan granule could regulate the expression levels of PI3K/Akt/FOXO3a pathway-related proteins in ovarian tissues, increasing the expression of PI3K and Akt proteins, and decreasing the expression of FOXO3a proteins.

## 3. MAPK Signaling Pathway

PTEN is involved in apoptosis through several signaling pathways, among which the activation of MAPK/ERK and PI3K/Akt signaling pathways is more common, and there are also interactions between PI3K/Akt and MAPK/ERK signaling pathways [22]; PTEN proteins can negatively regulate the activation of Raf1 by Ras in the MAPK/ERK pathway by activating Akt in the PI3K/Akt pathway, and can also directly negatively regulate Raf1 in the absence of Ras action, which in turn inhibits the biological effects of MAPK/ERK and promotes apoptosis.

MAPK pathway has an important role in inflammation, stress response, and apoptosis of cells. Among MAPK signaling pathways, extracellular signal-regulated kinase (ERK) regulates the inflammatory response and also regulates the stem cell factor (SCF)/tyrosine kinase receptor (c-kit) signaling pathway [23]. The MAPK pathway regulates apoptosis by a complex mechanism [24], at least through the following pathways: enhancement of c-Myc expression, phosphorylation of P53, involvement in Fas/Fasl-mediated apoptosis, activation of c-jun and c-fos, and induction of Bax translocation. In addition to the above five pathways, p38 MAPK can also induce apoptosis by enhancing TNF expression.

### 3.1. ER/C-MYC/TERT Signaling Pathway

Estrogen can regulate the expression of the TERT gene. c-Myc is the target gene of the estrogen receptor (ER). Estrogen binding to ER promotes the expression of transcription factor c-Myc. c-Myc can bind directly to the E-box at the 5′ end of the core promoter of the TERT gene of many cellular telomerases, which promotes TERT gene transcription, thereby activating telomerase and maintaining normal cellular function [25–27].

A randomized controlled trial [28] conducted by Chen found that Bushen Jianpi decoction was 93.30% effective in treating POI. Wang et al.[29, 30] observed that by increasing *E*_2_ levels, promoting ER activation, and stimulating c-Myc expression, Bushen Jianpi decoction can increase ovarian telomerase activity and telomere length, which in turn regulates TERT expression, thereby promoting proliferation and development of ovarian granulosa cells and maturation of oocytes.

### 3.2. P53

P53, as an oncogene, is located in the nucleus and can bind specifically to DNA, which can be activated when DNA is damaged, causing cells to be blocked in the *G*_1_ phase, and if the damaged DNA cannot be repaired, P53 can contribute to the apoptosis of damaged cells, and high expression of P53 heralds the cessation of cell growth or apoptosis [31].

A randomized controlled trial [32] carried out by Yanjin et al. found that the effective rate of Bushen Tiaochong decoction in treating POI reached 97.90%. Zhang [33] observed that the mechanism of Bushen Tiaochong decoction mainly can significantly improve the sex hormone level in mice, significantly increase the level of *E*_2_ and AMH, and decrease the level of FSH and LH; downregulate the expression of P53, while upregulate the expression of GnRHR, prolong the time of apoptosis, reduce the occurrence of follicular atresia, improve the reserve capacity of ovarian receptors, and then, coordinate ovarian function.

### 3.3. Ki67/ERK

Ki67 protein is expressed in the nucleus, is closely associated with mitosis, and plays an important role in cell proliferation [34].

A randomized controlled trial [35] conducted by Wu found that the overall effective rate of Bushen Huoxue decoction in treating POI was 93.33%. Zonghui [36] found that Bushen Huoxue decoction increased p-ERK1/2 protein levels in the ovarian tissue of aged mice, activated ERK1/2 phosphorylation, further improved follicular development in mice with decreased ovarian reserve function at advanced age, and increased the proliferation of follicular granulosa cells and granulosa cells of the oocyte complex.

### 3.4. p-38/Fas/FasL

The Fas/FasL pathway, also known as the death receptor pathway, acts as an apoptotic signaling receptor, forming a death-inducing complex by binding to its ligand FasL and activating its downstream caspase-3 to induce apoptosis [37].

Chunling [38, 39] showed that the Kuntai capsule could repair pathological damage to ovarian function in fertile rats, regulate serum sex hormone levels in mice with POF, downregulate FSH and LH levels, FasL protein, and mRNA expression, upregulate *E*_2_ and AMH levels, and Fas protein mRNA expression, and increase Fas mRNA expression and FasL mRNA expression to increase Fas mRNA expression and decrease FasL mRNA expression, thus protecting and improving ovarian function. In addition, the Kuntai capsule can improve the reproductive function of mice and increase the conception rate and pregnancy rate of mice with POF, and has no significant teratogenicity to the offspring mice.

Dan [40] found that the Gui Zhi Fu Ling capsule could significantly improve sex hormone levels in mice with POF, with the best effect in the middle dose group, which may be related to the inhibition of the Fas/FasL signaling pathway and reduction of ovarian cell apoptosis.

### 3.5. SCF

Stem cell factor (SCF), also known as Kit ligand, is a granulocyte-derived growth factor that binds to the oocyte c-Kit receptor and its signal is transduced through the PI3K channel.

Sun et al.[41] found that Zuo Gui pill upregulated Cx43 mRNA and protein expression in ovarian tissues of CTX-induced POF mice, increased the distribution of Cx43 between follicles and granulosa cells, and improved gap junction function.

Xinpeng [42] found that Bushen Tiaochong decoction promoted ovulation by increasing the sensitivity of ovaries to gonadotropins; by upregulating the expression of Cx-37 and downregulating the expression of SCF, it promoted the growth and development of early follicles and improved the gap junction function of ovarian tissues in rats and thus repaired ovarian functional damage. Xiang [43] found that Kun Bao pill reduced ovarian fibrosis by decreasing the expression of CTGF, TGF-*β*1, and SCF, which showed that Kun Bao pill had a positive intervention effect on POF induced by cisplatin injection in mice.

## 4. TGF-*β*/Smads Signaling Pathway

TGF-*β*/Smads signaling is an important transduction pathway that regulates follicular development, and abnormalities in either process of the transduction pathway may cause signaling disorders, leading to impaired follicular recruitment, inhibition of follicular growth and development, accelerated follicular atresia, and premature ovarian failure.

A randomized controlled trial [44] conducted by Liu Jia found that the total effective rate after treatment was 92.68% in the observation group and 81.71% in the control group when the observation group was given the combination of Siwu mixture combined with hexestrol and medroxyprogesterone acetate. Hongbo [45] found that Smad2/3 protein is an upstream regulatory signaling protein of Cyp19a1 through experiments, and by detecting Smad2/3 protein and its phosphorylated protein PSmad2/3, it was found that Siwu mixture upregulated Cyp19a1 expression by promoting the expression of Smad2/3, a Cyp19a1 regulatory protein.

Yameng [46] found that the Kuntai capsule could not only reduce the levels of sex hormones FSH and LH, increase the levels of *E*_2_ and AMH, repair the damaged ovarian tissue structure, improve ovarian blood supply, promote the development of rats follicles, reduce follicular atresia, and increase the number of mature follicles present, but also increase the expression of GDF-9 and EGR-1 protein and mRNA in rats ovaries. Chen [47] found that the Kuntai capsule may increase the expression of FSHR in rats' ovarian tissue by upregulating the expression of Smad2/3, improve the responsiveness of ovaries to FSH, promote follicle development, and reduce the level of serum FSH; meanwhile, it downregulates the expression of Smad7 in rats ovarian tissue to reduce follicle apoptosis, maintain follicle growth and development, and improve ovarian function in rats.

Zhu [48] found that Zuo Gui pill could upregulate the protein expression levels of ovarian GDF-9 and its signaling protein Smad2 in POF mice and promote the development of growing follicles in Smad2 mice. Compared with the model group, the ovarian GDF-9 and Smad2 protein expression increased and the ratio of ovarian growth follicles increased in the Zuo Gui pill group, suggesting that Zuo Gui pill may regulate ovarian function by improving the regulation of GDF-9/Smad2 signaling, thereby promoting the recruitment of initiating follicles, promoting follicular development, and inhibiting follicular atresia.

In addition, Yu [49] found that TCM tonic kidney and filling essence method could activate the Bmps/Smad signaling pathway, thus initiating primordial follicle development, inhibiting oocyte apoptosis, and improving ovarian function. Huiping [50] found that Bushen Huoxue decoction not only regulated follicle development and promoted granulosa cell proliferation related to the ActA/Smads pathway, but also promoted estradiol *E*_2_ secretion through the TGF-*β*1/Smads pathway to improve the local microenvironment of the ovary.

## 5. NF-KB Signaling Pathway

The NF-kB family plays an important role in physiopathological processes such as inflammation and immune response, oxidative stress response, cell proliferation, and apoptosis by regulating the expression of various pro-inflammatory factors, growth factors, and adhesion molecules. It has been reported [51] that NF-kB induces the expression of several pro-inflammatory factors, such as TNF-*α*, IL-*β*, FGF, VFGF, CINC1, and ICAM1.

### 5.1. The TNF-*α*

TNF-*α* is a multireactive cytokine that induces apoptosis of granulosa cells or early follicles by autocrine or paracrine means, and also causes vascular endothelial damage and inhibits hormone secretion and follicle growth and development.

In the rats with POF, the protein and gene expression of TNF-*α* and IFN-*γ* were increased in ovarian tissues, and IFN-*γ* could induce enhanced expression of MHC antigens on granulosa cells and activate a series of cytokines such as IL-1, IL-2, TGF-*β*, TNF-*α*, and FGF to produce autoimmune responses to cause follicular atresia. TNF-*α* can cause vascular endothelial damage and affect local blood flow in the ovary, which can block hormone secretion and follicular growth and development at all levels. After the intervention of renal tonic drugs, the expression levels of TNF-*α* and IFN-*γ* decreased, the expression of Bcl-2 protein increased, the expression of Bax protein decreased, and the apoptosis of granulosa cells was inhibited.

Zhou [52] observed that Erxian decoction could antagonize inflammatory symptoms in a dose-dependent manner in rats with POF, and could promote the secretion of vascular growth factors associated with POF and enhance ovarian reserve function.

Liu et al.[53] found that Cistanche can reduce follicular atresia and apoptosis by regulating sex hormone levels and inhibiting the expression of TNF-*α* and IFN-*γ* in rats, thus slowing down ovarian failure; Cistanche can also upregulate Bcl-2/Bax, suggesting that Cistanche has an inhibitory effect on POF, and the mechanism may be related to ovarian sex hormone levels, TNF-*α*, IFN-*γ,* and apoptosis-related protein Bcl-2/Bax expression.

Lan et al. [54] found that the Chinese herbal Fufang Yiqi Yangrong Fujing formula could effectively regulate serum LH, FSH, and E2 levels in CTX-induced POF mice and improve pituitary and ovarian endocrine functions. It could also increase the expression levels of serum IL-2 and TNF-*α*, inhibit the apoptosis of ovarian granulosa cells, restore ovarian function, and enhance ovarian reserve capacity.

### 5.2. VEGF and bFGF

Ovarian blood flow is an important factor in maintaining follicular growth, steroid hormone secretion, and follicular sensitivity to gonadotropins. The VEGF and bFGF are vascular endothelial growth factors, which can repair damaged follicles and improve damaged ovarian vascular permeability and can specifically promote cell proliferation survival and chemotaxis in steroid hormone-producing organs and promote neovascularization. The bFGF plays an important role in luteinizing, mainly in promoting the growth and development of follicular corpus luteum, and also in providing nutrition to the corpus luteum entity.

Xu [55] found that Bushen *Tiaochong decoc*tion could prevent the occurrence of premature ovarian failure in rats, and its mechanism of action might be related to the positive effect of certain components in Chinese medicine in the enhancement of gonadotropins, which promotes the repair of ovarian function and improves ovarian function. Serum FSH and LH were decreased, and *E*_2_ was increased in rats with premature ovarian failure by Chinese medicine gavage, and the expression of the VEGF and the bFGF in ovarian tissues was increased [56], and the expression of TNF-*α* and IFN-*γ* was downregulated to reduce follicular atresia and slow down the depletion of follicles.

In addition, the expression of VEGF and bFGF was significantly increased in rats with POF after gavage of Kuntai capsules (*p* < 0.05) [57]. This indicates that Kuntai capsules can protect vascular endothelial cells, smooth blood flow in the ovaries, improve ovarian reserve capacity, and prevent POF. By regulating hormone levels and upregulating the expression of VEGF and bFGF mRNA to alleviate the damage to ovarian function caused by Leigongteng polysaccharide tablets, it delayed or blocked POF, promoted follicle development, and improved ovarian function.

## 6. Keap1 Nrf2/ARE Pathways

Oxidative stress is one of the key factors leading to apoptosis of oocytes and ovarian granulosa cells. The key pathway for cellular resistance to oxidative stress [58] is the Kelch-like epichlorohydrin-associated protein 1 (Keap1)-nuclear factor E2-related factor 2 (Nrf2)/antioxidant response element (ARE), which initiates antioxidant enzymes downstream of the pathway, including superoxide dismutase (SOD), quinone oxidoreductase, glutathione peroxidase (GSH-Px), and catalase (CAT) [59].

A randomized controlled trial [60] conducted by Ma et al. found that in patients with POI infertility, the test group used Bushen Culuan decoction and the control group used “estradiol valerate tablets + clomiphene + progesterone,” and the results showed that the ovulation rate, pregnancy rate, sex hormone level, and TCM symptoms score improved significantly better in the test group than the control group. The total effective rate of treatment in the trial group was 95.35%. Bushen Culuan decoction ameliorated the oxidative stress induced by raffinose polysaccharide [61], decreased the content of ovarian DNA oxidative damage product 8-OHdG and lipid peroxidation product MDA, elevated the activity of ovarian CAT, GSH-PX, SOD, and HO-1 antioxidant enzymes, and inhibited Keap1, through the Nrf2/ARE signaling pathway, and Bach1 nuclear protein expression and promoted Nrf2 nuclear translocation, thus activating downstream antioxidant enzyme activities, which in turn attenuated the ovarian oxidative damage induced by raffinose polysaccharide.

Yu-Zhi [62] observed that Yiguan Jian decoction not only could improve ovarian morphology and ovarian quality in a rat model of POF, but also could repair damaged and protect normal ovarian cells by mobilizing T-SOD and CAT, thus reducing the damage to ovarian cells by peroxidation-related substances such as MDA and caspase-3.

## 7. Ovarian Silencing Regulatory Proteins (SIRTs)

SIRTs are regulatory factors involved in the aging process. Early studies suggested [63] that SIRTl promotes follicle development, improves ovarian reserve function, and prolongs ovarian lifespan. SIRT1 inhibits the NF-KB inflammatory signaling pathway and reduces inflammatory factor release. It increases the expression of the anti-apoptotic protein Bcl-xl and downregulates the pro-apoptotic proteins caspase-3 and Bax, through the FOXO1 signaling pathway, and inhibits apoptosis.

Tong et al. [64] found that Zuo Gui pill and You Gui pill could increase follicle count, SIRT1, and serum AMH and INHB, and decrease serum LH and FSH concentrations in mice with POF, in addition to the fact that the number of primordial follicles in the You Gui pill group was significantly higher than that in the Zuo Gui pill group, indicating that Zuo Gui pill and You Gui pill had significant anti-ovarian aging effects, and their mechanism of action was related to the upregulation of ovarian SIRT1 expression.

The effects of single herbs and Chinese herbal formulas on the regulation of the POI signaling pathway are summarized in Tables 1 and 2.

## 8. Conclusion

Signaling pathways are used as enzymatic response pathways that can transmit molecular signals from outside the cell to the cell in order to function, and the pathogenesis of various diseases involves the participation of related signaling pathways. In recent years, research on TCM interventions in related signaling pathways has been on the rise, especially in TCM to further understand the pathogenesis of POI by studying interventions in the transmission of related signaling pathways. There are numerous pathways related to two major factors of POI: genetics and immunity. PI3K/Akt signaling pathway, TGF-*β*/Smads signaling pathway, and MAPK signaling pathway also restore ovarian function by regulating apoptosis, oxidative stress response, etc. In conclusion, Chinese herbal medicines alone or in combination can affect the factors related to the development of POI (granulosa cell apoptosis, ovarian blood supply, ovarian reserve, ovarian oxidative damage, gap junctions, ovarian fibrosis, follicular development, follicular atresia, and other biological processes) by regulating one or more signaling pathways, thus playing a role in antioxidative stress, preventing, and controlling the side effects of chemotherapy, protecting ovarian function, controlling the onset of aging, and improving ovarian reserve function. However, most of the current studies on signaling pathways related to TCM interventions are in their infancy, with relatively few studies and uncertain clinical efficacy. Therefore, further in-depth clinical studies are needed in the future, close to the clinic, to provide useful methods for the clinical treatment of POI patients.

## Figures and Tables

**Table 1:** The regulatory effects of Traditional Chinese medicine on signal pathways related to POI.

Chinese herbal	Sources	Classification	Efficacies	Pathways	Targets	Experimental model	Roles
Ginsenoside Rg1 [10]	Ginseng	Qi tonics	It is a great tonic for the vital energy, restores the pulse, and fixes the detachment, tonifies the spleen, benefits the lung, generates fluid and nourishes the blood, and calms the mind.	PI3K/Akt/mTOR signaling pathways	PI3K↓, Akt↓, mTOR↓, S6k↓	SPF-grade female BALB/*c* mice	Activation of autophagy in ovarian tissues to inhibit the onset of aging.

Epimedium glycoside [11]	Epimedium	Yang tonics	Tonifying the kidney and Yang, strengthening the muscles and bones, dispelling wind and dampness.	PI3K/Akt/mTOR signaling pathways	PI3K/Akt/mTOR↑	Clean-grade female uncrossed Wistar rats	Inhibit oxidative stress and reduces tissue apoptosis.

Cistanche [53]	The fleshy stems of Cistanche or Cistanche, Cistanche fannii, etc., of the family Cistanaceae.	Yang tonics	Tonifying the kidney and Yang, benefiting the essence and blood, moistening the intestines, and opening the bowels.	NF-kB signaling pathways	TNF-*α*↓, IFN-*γ*↓, Bcl-2↑, Bax↓	SPF-grade 12-week-old SD female rats	Reduce follicular atresia and apoptosis, which in turn slows ovarian failure.

**Table 2:** The regulatory effects of Chinese herbal formula on signal pathways related to POI

Recipe	Compositions	Classification	Efficacies	Pathways	Targets	Experimental model	Roles
Yulinzhu [6]	Radix Angelicae Sinensis, Radix Rehmanniae Praeparata, Semen Cuscutae, ginseng, branched Atractylodes macrocephala, Poria, Radix Paeoniae Alba, Cortex Eucommiae, Zanthoxylum piperitum. Rhizoma Ligustici, Radix Glycyrrhizae	Tonic prescriptions	Warming the kidneys and strengthening the spleen to produce essence	PI3K/Akt/mTOR signaling pathways	TSC1↓, TSC2↓, Rheb↑, P-s6k1↑, P-4e-bp1	SPF BALB/*c* female mice with normal motility cycles at 6 to 8 weeks of age.	It can inhibit microenvironmental oxidative stress.

Jiajian Guishen pill [8]	Semen Cuscutae, semen spleen, Radix Rehmanniae, Radix Rehmanniae, Radix Angelicae Sinensis, Radix Paeoniae Alba, Salviae miltiorrhiza	Tonic prescriptions	Tonifying the kidney, strengthening the spleen, tonifying the liver, and invigorating the blood	PI3K/Akt/mTOR signaling pathway	PI3K↑, Akt↑, mTOR mRNA↑	SPF ICR female mice.	Improve ovarian reserve function and increase the number of follicles.

Xianzi Yizhen capsule [9]	Radix Rehmanniae Praeparata, Radix et Rhizoma Polygonati, Radix et Rhizoma Drynariae, Radix et Rhizoma Continuum, Semen Cuscutae, semen spleen	Tonic prescriptions	Tonifying the kidney and filling the essence	PI3K/Akt/mTOR signaling pathways	Ki67↑, Akt↑, PI3K↑	SPF female C57BL/6J type mice.	Increase the content of primordial follicles, secondary follicles and sinus follicles, and decrease the content of atretic follicles.

Guiluo's Anzang decoction [12]	Radix Rehmanniae Praeparata, Fructus Fritillariae, Semen Cuscutae, Radix et Rhizoma Polygoni, Paeoniae Alba	Tonic prescriptions	Nourishing Yin, tonifying the kidneys, calming the mind, and relieving irritability	Bax/CytC/Caspase-3 signaling pathways	Bcl-2↑, Bax↓	SPF healthy female SD rats	Reduce granulocyte apoptosis and increase granulocyte secretion.

Kuntai capsule [14, 38, 39, 46, 47, 57]	Radix Rehmanniae Praeparata, Rhizoma Polygonati, Radix Paeoniae Alba, Radix Scutellariae Praeparata, Radix Aconiti, Poria	Tonic prescriptions	Nourishing Yin, clearing heat, calming the mind, and relieving irritability	Bax/CytC/Caspase-3 signaling pathways, p-38/Fas/FasL signaling pathways, TGF-*β*/Smads signaling pathways, NF-kB signaling pathways	Bcl-2↑, Bcl-xl↑, Bax↓, Bad↓, Fas mRNA↑, FasL mRNA↓, GDF-9↑, EGR-1↑, Smad7↓, VEGF↑, bFGF↑	SPF healthy female SD rats	Maintain the balance between pro-apoptotic and anti-apoptotic proteins and improve ovarian reserve function; improve ovarian blood supply, promote follicle development, reduce follicular atresia and increase the number of mature follicles present in rats.

Yangyin Shugan granule [15]	Radix Bupleurum, Radix Paeoniae Alba, etc.	Mediative formulas	Nourishing Yin and soothing the liver	Bax/CytC/Caspase-3 signaling pathways	Bcl-2↑, Bax↓, Caspase-3↓, FOXO3a↓	SPF healthy female SD rats	It can inhibit apoptosis.

Zuogui pill [17, 18, 21, 41, 48, 64]	Radix Rehmanniae Praeparata, Rhizoma Dioscoreae, Fructus Lycii, Cornu Cervi Pantotrichum, Radix Achyranthes Bidentatae, Semen Cuscutae, antler gum, turtle board gum	Tonic prescriptions	Nourishing Yin, tonifying the kidney, and nourishing the blood	Bax/CytC/Caspase-3 signaling pathways, FOXO3, SCF, TGF-*β*/Smads signaling pathways	Bcl-2 mRNA↑, Bax↓, FOXO3a↓, CTX↑, Cx43 mRNA↑, Smad2↑, GDF-9↑	Human ovarian granulosa cells; SPF 8-week-old BALB/*c* female mice	It can inhibit chemotherapy-induced granulosa cell apoptosis and protect ovarian function; improve suture junctions; promote recruitment of initiating follicles, promote follicular development, inhibit follicular atresia, and regulate ovarian function.

Erxian decoction [20, 52]	Herba dipteris, Epimedium herba, Phellodendron phellodendron, Euphorbia officinalis, Angelica, Anemone anemone	Tonic prescriptions	Warming kidney Yang, tonifying kidney essence, and dipping kidney fire	FOXO3 transcription factor -P27/Bim	FOXO3↓, P27KiPi↓, Bim↓	Clean-grade SD healthy female rats	Promote granulosa cell proliferation and inhibit granulosa cell regulation; promote the secretion of vascular growth factor associated with premature ovarian failure in rats, and enhance ovarian reserve function.
Bushen Jianpi decoction [29, 30]	Polygonatum officinale, Radix et Rhizoma Polygonatum, Radix et Rhizoma Polygonatum, Fructus Lycii, Atractylodes Macrocephala, Poria	Tonic prescriptions	Tonifying the kidneys and strengthening the spleen	ER/c-myc/TERT signaling pathways	c-Myc↑, TERT↑	B6AF1 female mice	It can promote the proliferation and development of ovarian granulosa cells and the maturation of oocytes.

Bushen Tiaochong decoction [33, 42, 55]	Cuscuta seed, Euphorbia officinalis, Ripe Rehmannia, Cistanche, yellow essence, amethyst, Schisandra fruit, Angelica, Ligusticum wallichii, etc	Tonic prescriptions	Tonifying the kidneys and regulating the flushing process	P53, SCF, NF-kB signaling pathways	P53↓, GnRHR↑, Cx-37↑, SCF↓, VEGF↑, bFGF↑, TNF-*α*↓, IFN-*γ*↓	Clean-grade female SD rats	Prolong the time of apoptosis, reduce the occurrence of follicular atresia, improve the reserve capacity of ovarian receptors and thus coordinate ovarian function; promote the growth and development of early follicles, improve the function of ovarian tissue gap junctions and thus repair ovarian function damage in rats.

Bushen Huoxue decoction [36, 50]	Herba epimedium, Semen Cuscutae, Fructus Lycii, Fructus Lycii, Fructus Morindae, mulberry, raspberry, yam, Radix Codonopsis, Radix Astragali, Radix Paeoniae Alba, Fructus Ulmoides, bark, Salviae Miltiorrhiza, Radix Angelicae Sinensis, Radix Angelicae Sinensis	Tonic prescriptions	Tonifying the kidney and invigorating the blood	Ki67/ERK	p-ERK1/2↑, ERK1/2↑	Mouse intrasinus follicular granulosa cells	It can improve follicular development and increase the proliferation of follicular granulosa cells and granulosa cells of the oocyte complex in mice with reduced ovarian reserve function at an advanced age.

Gui Zhi Fu Ling capsule [40]	Cassia twig, Poria cocos, peony bark, peony root, peach kernel	Blood-regulating formula	Promoting blood circulation, removing blood stasis, and eliminating symptoms	p-38/Fas/FasL	Fas/FasL↓	SPF female Wistar rats	Reduce ovarian apoptosis.

Kun Bao pill [43]	Chasteberry, raspberry, Cuscuta, etc.	Tonic prescriptions	Nourishing the liver and kidneys, calming and tranquilizing the mind, nourishing the blood, and opening the meridians	SCF, TGF-*β*	CTGF↓, TGF-*β*1↓, SCF↓	SPF healthy female SD rats	Reduce ovarian fibrosis.

Siwu mixture [45]	Radix Rehmanniae Praeparata, Radix Angelicae Sinensis, Radix Paeoniae Alba, Ligustici wallichii	Tonic prescriptions	Nourishing Yin and replenishing blood	TGF-*β*/Smads signaling pathways	Smad2/3↑, Cyp19a1↑	Healthy female SD rats	It can promote follicular growth and development and slow down follicular atresia.

Yiqi Yangrong Fujing formula [54]	Astragalus, Bacopa monnieri, Dendrobium Ferrugineum, Rhizoma Polygonatum	Tonic prescriptions	Benefiting Qi, warming Yang, nourishing Yin, and restoring essence	NF-kB signaling pathways	IL-2↑, TNF-*α*↑	Healthy female C57BL/6 mice	Inhibit the apoptosis of ovarian granulosa cells, restore ovarian function, and enhance ovarian reserve capacity.

Bushen Culuan formula [61]	Radix chasteberry, Semen Cuscutae, Fructus Lycii, Radix et Rhizoma mulberry, Radix et Rhizoma Sequoiae, Radix Angelicae Sinensis, Radix Paeoniae Alba, Radix Zelenium	Tonic prescriptions	Tonifies the kidneys and enhances the essence	Bax/CytC/Caspase-3 signaling pathways, Keap1/Nrf2/ARE signaling pathways	Akt↓, mTOR mRNA↓, PI3K mRNA↓, Bcl-2↑, Keap1↓, Bach1↓	SPF 8-week-old female BALB/*c* mice	Reverse excessive apoptosis of granulosa cells, reduce follicular atresia, reduce excessive activation of primordial follicles, and protect ovarian reserve; reduce ovarian oxidative damage.

Yiguan Jian decoction [62]	Raw Rehmanniae, Radix Aristophanae, Angelica, Wolfberry, chinaberry	Tonic prescriptions	Nourishing Yin and softening the liver	Keap1/Nrf2/ARE signaling pathways	T-SOD↑, CAT↑, MDA↓, Caspase-3↓	SPF healthy female SD rats	Protect normal ovarian cells.

## Data Availability

The data that support the findings of this study can be obtained from the corresponding author upon reasonable request.
